# The Application of Nurse Stratified Management in Nursing Management

This article has been retracted.

**DOI:** 10.1155/2022/6368765

**Published:** 2022-07-22

**Authors:** Qing Liu, Yujuan Guo, Pin Wei, Chao Cui

**Affiliations:** ^1^Hemodialysis Room, Chengyang District People's Hospital, Qingdao, Shandong, China; ^2^Obstetrics Department, Chengyang District People's Hospital, Qingdao, Shandong, China; ^3^Blood Purification Center, Qingdao Municipal Hospital, Qingdao, Shandong, China

## Abstract

**Objective:**

To explore the application value of nurse stratified management in nursing management.

**Methods:**

One hundred nurses who worked in our hospital from June 2019 to September 2021 were recruited and assigned via the random number table method to an observation group (*n* = 50) and the control group (*n* = 50). The control group received routine nursing management, and the experimental group received stratified nursing management. The nursing quality, practice happiness, error rate, patient complaint, and patient satisfaction were compared between the two groups.

**Results:**

The experimental group showed a significantly higher nursing quality than the control group (*P* < 0.05). The experimental group had significantly higher practice happiness among nurses than the control group (*P* < 0.05). Stratified nursing management mode resulted in a significantly lower error rate and patient complaint versus routine nursing management mode (*P* < 0.05). Patients were more satisfied with stratified nursing management than with the routine nursing management (*P* < 0.05).

**Conclusion:**

The nurse stratified management method effectively improves the nursing quality and practice happiness of nurses, reduces the error rate of nursing and patient complaint, and increases nursing satisfaction.

## 1. Introduction

In recent years, with the continuous advancement of medical technology, patients have increasingly higher demands for nursing quality [1]. Hospital nursing quality is an important manifestation of a hospital's comprehensive ability, the improvement of which depends on strict nursing management. The use of nursing management in daily nursing provides patients with the highest quality nursing services [2], which benefits clinical treatment efficiency and patient nursing satisfaction. Nursing hierarchical management is a new nursing management model [3] that clarifies the responsibilities of nurses to maximize the utilization of nursing resources and fully motivate the nurses, which provides patients with the finest nursing services and increases the satisfaction of patients with clinical care [4]. Fang et al. [5] revealed that the stratified nursing management model improved the quality of patient care. One hundred nurses at our hospital from June 2019 to September 2021 were recruited to explore the effects of stratified care management.

## 2. Materials and Methods

### 2.1. Study Population

One hundred nurses who worked in our hospital from June 2019 to September 2021 were recruited and assigned via the random number table method to an observation group (*n* = 50) and the control group (*n* = 50). Undersigned informed consent was obtained prior to enrollment in this study. The study protocol was approved by the hospital ethics committee, and all processes complied with the Declaration of Helsinki ethical guidelines for clinical research. The ethics number is XTQ20190617.

All nurses were informed about the study and participated voluntarily. The control group included 4 male nurses and 46 female nurses, aged 21–38 (27.63 ± 1.23) years, with a working year of 2–13 (6.82 ± 1.13) years. There were 5 male nurses and 45 female nurses in the experimental group, aged from 22 to 38 (27.73 ± 1.28) years, with a working year of 3–14 (7.12 ± 1.06) years. There was no significant difference in the general data of nurses between the two groups, as shown in Table 1. The flow chart is in Figure 1.

### 2.2. Methods

The nurses in the control group received routine nursing management, and the nurses in the experimental group received the nursing stratification nursing management. (1) The stratification of nursing incorporated the specific conditions of hospital management establishes a stratification mechanism for nurses, designates or dismisses responsible nursing team leaders through job competition, and stratifies the nurses based on their clinical experience, academic qualifications, and professional titles. The head nurse was responsible for the organization, and the members of the group discussed and formulated the nursing responsibility stratification system [6]. (2) Relevant nurses are required to provide continuous nursing services and guidance, closely monitored the patient's condition, and offered health education. In addition, the senior nursing staff is also responsible for supervising, managing, and guiding the implementation and practice of daily nursing work by subordinate nursing staff. The primary responsibility of the responsible team leader is to supervise the care of elderly or critically ill patients and train junior nurses [7]. (3) Hierarchical nursing management was implemented based on the ability of nurses to obtain more satisfactory nursing services and better nursing quality. With reference to nurses' clinical experience and educational level, hospitals categorize and implement nursing tasks, optimize human resource allocation, and correctly construct and improve the specific content and process of nursing work, thereby enhancing nursing quality [8]. (4) A management system in line with nursing hierarchical management was established, and specific training programs and assessment standards and reasonable training and assessment systems were formulated based on the specific conditions of each department. The level training was completed through the corresponding subitems and groups. The nursing staff was trained by on-site teaching or nursing special lectures, to fully combine theoretical knowledge with practical experience, thereby enhancing the nursing quality. Nurses maximize their professional nursing level and ability when conducting ward rounds and patient consultations. A corresponding reward and punishment system was established to promote nursing staff to improve their initiative and enthusiasm for nursing work, which consequently improved patient care satisfaction and nursing quality [9].

### 2.3. Control Indicators

1. Nursing quality: the nursing was evaluated using a self-made scale in our hospital. The evaluation content included four aspects as follows: basic nursing, health education, overall nursing, and ward management. The total score for each aspect was 100 points, and the higher the score, the better the quality of care.
2. Nurse happiness: the self-made nurse happiness scale was used for evaluation. The total score on the scale was 100 points. The higher the score, the stronger the nurse's happiness.
3. Nurse error rate: it was recorded by the relevant supervisors in our hospital. Nurse error rate = the number of nurses with errors/total number of nurses.
4. Patient complaint rate: it was recorded by the relevant medical staff in our hospital.
5. Patient satisfaction: a self-made satisfaction survey questionnaire was used in our hospital to investigate the satisfaction degree of the patients with the responsible nurses. The full score is 100 points, 80 points and above indicate highly satisfied, 60-79 points indicate satisfied, and a score of 59 and below indicates dissatisfied. Total patient satisfaction = (highly satisfied  + satisfied) number of cases/total number of cases × 100%.

### 2.4. Statistical Analysis

Data were expressed as the mean ± standard deviation. Statistical analysis was performed using the SPSS 22.0 (IBM, Armonk, NY, USA). Differences in measurement data expressed as (*x* ± *s*) and count data expressed as the number of cases (rate) were compared using the Student's *t*-test and the Chi-square test. *P* < 0.05 was set as the cut-off for statistical significance. The GraphPad Prism8 was used for graphics rendering.

## 3. Results

### 3.1. Nursing Quality

Table 2 shows a significantly higher nursing quality of the nurses in the experimental group when compared with the control group (*P* < 0.05).

### 3.2. Happiness of Nurse Practitioners

The experimental group had significantly higher happiness in practice than the control group (*P* < 0.05), as shown in Figure 2.

### 3.3. Nurse Error Rates

Stratified nursing resulted in a significantly lower error rate for the nurses than for the control group (*P* < 0.05, Table 3).

### 3.4. Patient Complaint Rates

The nursing management model in the experimental group resulted in a significantly lower patient complaint rate than routine management in the control group (*P* < 0.05, Table 4).

### 3.5. Patient Satisfaction

Patients were more satisfied with the stratified nursing versus the routine nursing (*P* < 0.05, Table 5).

## 4. Discussion

Currently, there exist numerous issues in the nursing work in most hospitals, such as the uneven distribution of human resources and the pressure on nursing work, which downgrades the quality of nursing in hospitals [10]. Zhang et al. [11] have found that a scientific and effective management model for nursing staff contributed to improving nurses' sense of responsibility and mobilizing their enthusiasm for work which effectively ensures the integrity and continuity of nursing [12]. In traditional nursing management, the inconsistency of nursing quality due to the individual differences of nurses may result in poor nurse-patient relationships [13]. The stratified nursing management model clarifies the relevant responsibilities of nursing staff and fully utilizes the human resources of the hospital [14]. It compensates for the shortcomings of the conventional nursing management mode and maximally utilizes the abilities of nurses [15]. Xu and Lei standardized the implementation of TCM nursing programs on the basis of the single-patient management model and improved the management content using hierarchical management and process control, which highlighted the nursing characteristics of TCM hepatology and reduced nursing errors [16]. In addition, the stratified nursing management avoids the blindness of nursing, thus reducing the work difficulty of primary nurses and ensuring the safety of clinical nursing [17].

The results of this study showed higher nursing quality in the experimental group than in the control group. The reason may be that the hierarchical management model of nurses has complete training and guidance that ensured standardized nursing methods and outcomes [18]. Moreover, the nurses in the experimental group had significantly higher practice happiness and a better sense of well-being in practice, which may be attributed to the fact that the hierarchical management model allowed a better performance of the nurses through the reasonable assignment of nursing work by evaluating their ability, which facilitates the self-realization of the nurses [19]. Furthermore, the experimental group had a lower error rate and patient complaint rate, and a higher patient satisfaction rate than the control group, which indicates that the hierarchical management model of nurses effectively reduced the clinical error rate of nurses, thereby reducing the complaints of patients and improving patient satisfaction [20]. The possible explanation is that the hierarchical management model of nurses clarifies the process and content of nursing for the nurses, which contributes to avoiding nursing mistakes and inaccuracy [21].

Despite numerous studies on the quality of care in hospitals [22, 23], this study concentrated on efficient assessment and enhanced management and provided guidance and assessment methods based on the results of this study to offer valid clinical evidence for improving the quality of care in hospitals.

The limitations of this study are the small sample size and short follow-up duration. Future studies with larger sample size and long follow-up duration will be conducted to provide more clinical evidence.

To sum up, the nurse stratified management method effectively improves the nursing quality and practice happiness of nurses, reduces the error rate of nursing and patient complaint, and increases nursing satisfaction.

## Figures and Tables

**Figure 1:** Research flow chart.

**Figure 2:** Comparison of nurse practitioner happiness (*x* *±* *s*). Note: ^*∗*^*P* < 0.05.

**Table 1:** Comparison of general data of patients (*n* (%)).

	Control group (*n* = 50)	Experimental group (*n* = 50)	T/*x*^2^	*P*
Gender			0.122	0.727
Male	4	5		
Female	46	45		
Mean age (year)	27.63 ± 1.23	27.73 ± 1.28	−0.398	0.691
Mean working year (year)	6.82 ± 1.13	7.12 ± 1.06	−1.369	0.174

**Table 2:** Comparison of nursing quality (*x* ± *s*).

Groups	*n*	Basic care	Health education	Holistic care	Ward management
Control group	50	94.21 ± 2.35	93.46 ± 2.47	94.11 ± 2.69	93.44 ± 3.10
Experimental group	50	87.91 ± 2.28	88.12 ± 2.39	87.58 ± 2.35	88.92 ± 2.93
*X * ^2^	—	13.605	10.986	12.927	7.493
*P*	—	<0.001	<0.001	<0.001	<0.001

**Table 3:** Comparison of nurse error rates (*n* (%)).

Groups	*n*	Number of nurses with errors	Number of nurses without errors	Error rate
Control group	50	14	36	14 (28%)
Experimental group	50	2	48	2 (4%)
*t*	—	—	—	10.714
*P*	—	—	—	0.001

**Table 4:** Comparison of patient complaint rates (*n* (%)).

Groups	*n*	Complaints	Noncomplaint	Complaint rate
Control group	50	12	38	12 (24%)
Experimental group	50	1	49	1 (2%)
*t*	—	—	—	10.698
*P*	—	—	—	0.001

**Table 5:** Comparison of patient satisfaction (*n* (%)).

Groups	*n*	Very satisfied	Satisfied	Dissatisfied	Total
Control group	50	11	21	18	32 (64%)
Experimental group	50	29	17	4	46 (92%)
*t*	—	—	—	—	11.422
*P*	—	—	—	—	0.001

## Data Availability

No data were used to support this study.
